The article "Analysis and Research on Influencing Factors of College Students' Satisfaction with Physical Education" was retracted in 2023. Reasons: signs of a paper mill; suspected computer-generated content; unreliable results or conclusions; concerns about the data.

# Analysis and Research on Influencing Factors of College Students' Satisfaction with Physical Education

**DOI:** 10.1155/2022/7506157

**Published:** 2022-08-10

**Authors:** Xing Liu, Meiyin Dong, Yachen Li, Shanshan Gao, Minghui Ye

**Affiliations:** ^1^Guangzhou City University of Technology, Guangzhou 510800, China; ^2^Department of Physical Education,Shijiazhuang University, Shijiazhuang 050035, China; ^3^Guangdong Technology College, Zhaoqing 526100, China; ^4^Sports Training Department of Hebei Institute of Physical Education, Shijiazhuang 400067, China

## Abstract

Physical education is an important part of a university, and the satisfaction of college students for physical education directly determines the teaching effect of physical education. Therefore, it is of great significance to understand college students' satisfaction with physical education and its influencing factors for improving the level of physical education. In this paper, by means of multistage sampling, probability sampling according to scale and random equidistant sampling, 7 main campuses, including 36 subcampuses, are selected for data entry, cleaning, and calculation by using the college physical education teaching system. Through the investigation of 1752 students, the results show that there are significant differences in grade, gender, cognition, credit, sense of responsibility, and teaching content (*P* > 0.05), which are all factors affecting college students' satisfaction. Cognition, grades, credits, and make-up test rate are the main influencing factors, with the influence degree ranging from 1 to 3, and there are significant differences in OR value and *P* value. Therefore, in the process of physical education, we should pay attention to the above-mentioned influencing factors, effectively reduce the occurrence rate of make-up examination and reexamination, adjust unreasonable teaching content, and improve students' satisfaction with physical education.

## 1. Introduction

University is a key period to improve knowledge and physical quality, and reasonable physical exercise is needed Zapata-Lamana et al. [1]. Because the sports activities of college students in China are mainly spontaneous and supplemented by teaching, students cannot get enough exercise and get fewer sports credits Wang et al. [2]. According to the survey of sports centers and teaching centers in China, the physical education teaching rate of universities in Northeast China, Southeast China, and West China is 32.3%, Wang and Li [3], which is significantly lower than the survey requirements of the Ministry of Education for college students' physical exercise. Therefore, how to reasonably carry out physical education for students in remote areas has become the focus and hot spot of domestic scholars. Some scholars, Rojo-Ramos et al. [4], believe that the Ministry of Education put forward the “Methods for College Students' Physical Education,” which is a guiding method for college students' physical education and can improve the level of physical education. Some scholars, Ren and Shi [5], believe that “College Students' Physical Education Method” belongs to extensive research, lacks pertinence, and is not suitable for Northeast China, West China, and other regions. Based on the above reasons, this paper, with the support of the College Student Affairs Office, conducts a special investigation on college students' satisfaction with physical education, finds out the main influencing factors, and aims to find ways to improve college students' satisfaction with physical education. A satisfaction survey can improve the teaching effect by understanding the influencing factors and physical education teaching content. How to make a reasonable evaluation plan and find out the factors affecting teaching satisfaction is a problem that needs to be solved in college physical education at present. Some scholars believe that the classification of teaching content and sports effect makes the research results more accurate. However, the complexity of influencing factors of physical education and the lack of students' cognition of physical education make the effect of physical education poor. Some scholars believe that the premise of physical education is to find out the factors, so we should find out the internal influencing factors through the analysis of content and time and make a better physical education teaching plan. From the above comparative research results, we can see that foreign scholars have done more research on educational satisfaction, pay attention to the analysis of the influencing factors of satisfaction, and formulate relevant teaching strategies according to the influencing factors. However, Chinese scholars have less research on teaching satisfaction, especially on the factors of physical education teaching satisfaction. In addition, the foreign teaching satisfaction research is not suitable for the domestic education situation, so we should combine the domestic college physical education situation, carry out the corresponding satisfaction survey, find out the main influencing factors, and put forward the corresponding strategies. Therefore, some scholars put forward a variety of influencing factors of physical education, such as rerepair rate, content rationality, complexity, and teaching score. The specific results are shown in Table 1.

From Table 1, we can see that in the research on physical education satisfaction, graduate students have the highest satisfaction, followed by freshmen and finally, college girls. Among them, the complexity of physical education is the main aspect that affects satisfaction, followed by content, relevance, and so on. The data in Table 1 suggest that physical education satisfaction is influenced by many factors, such as subjective, objective, and other aspects. Therefore, improving physical education satisfaction is a complex research project that should be comprehensively analyzed from various aspects. Moreover, the satisfaction of physical education runs through the stages of college students and postgraduates, so it is the focus of physical education and the future research direction of physical education. Therefore, the analysis of the satisfaction degree of physical education teaching aims to formulate corresponding research strategies and improve the teaching level. Some scholars have theoretical analysis on the influencing factors of physical education and think that the premise of finding influencing factors is to improve the teaching level. However, there is a lack of quantitative analysis on the influencing factors such as capacity rationality, complexity, and teaching score. Based on this, through the comparison between the study group and the control group, this paper finds out the influencing factors of teaching satisfaction and improves the level of college physical education. The related research results are shown in Figure 1.

As can be seen from Figure 1, there are many influencing factors of physical education satisfaction, and the degree of influence is not the same. Therefore, it is necessary to carry out regression analysis on different influencing factors. Otherwise, it is difficult to find the main influencing factors accurately. The data in Figure 1 shows that there is a minimum area value in each index, and the minimum area value increases from left to right in turn, indicating that the significant role of the index is gradually exerted and the influence level is improved in turn. At the same time, each index has a maximum area value, and the area decreases from top to bottom, which shows that the convergence of the index is gradually enhanced, and the influence of the index is increasing day by day. Therefore, the indicators in Figure 1 show double analysis of influence depth and influence content, and the analysis of various influencing factors is deepening, and the influence scope is expanding. On this basis, this paper analyzes the influencing factors of college students' satisfaction, aiming to find the main influencing factors and provide support for the improvement of college physical education teaching level. This article aims at the sports teaching satisfaction question and carries on the correlation influence factor analysis; the concrete content includes the following: The first chapter carries on the analysis of this article's research background, the research significance, and the purpose, elaborating the sports teaching satisfaction proposed condition. The second chapter analyzes the research methods of this paper, including the general data, research methods, research contents, and research indicators of physical education satisfaction. The third chapter compares the research results of the observation group and the control group, discusses the teaching effect and the content of satisfaction grade, and obtains the corresponding comparison results. The fourth chapter discusses the influencing factors of physical education satisfaction and analyzes the functions and reasons of different factors combined with the corresponding research results. The fifth chapter summarizes the research results of this paper and discusses the shortcomings and future development trends of the research results of this paper.

## 2. Research Objects and Methods

### 2.1. Subjects of Study

According to the regulations in the Method of Physical Education for College Students put forward by the Ministry of Education, 1752 college students were selected as the research objects, and the parents were informed of the purpose, significance, and role of the research, as well as the possible dangers in the investigation process. Among them, 1742 students met the survey requirements, accounting for 85.4% of the total. The following are included in the survey requirements: (1) college students, sports scores below 65 points, or failed; (2) freshmen, and there is no major violation of discipline; (3) students who signed an informed consent form, which is approved by the Academic Affairs Office of our school; Exclusion criteria for the investigation requirements: (1) students who drop out of school; (2) students who do not cooperate with the investigation; (3) students who quit halfway or fail to follow the questionnaire survey.

### 2.2. Methods

The sampling method is a combination of probability perspective to size sampling (PPS) and random equidistant sampling. The sample size calculation method: Satisfaction rate of students' physical education before the investigation is 30%, satisfaction rate after measures is 54%, confidence level is 95% (*α* = 0.05), and test validity is 90% (*β* = 0.1). Assuming that the per capita sports score is *s*, the whole school sports score is ∑*s*, and the sports weight of any student is *w*_*i*_, the calculation of the inclusion probability is *p*. The result is shown in the following:

(1) $$\begin{array}{c} \left\{\begin{array}{c} p=\frac{s}{\sum s}\cdot w_{i},{\frac{1}{w}}_{i}=0,\\ p^{\prime }=s\cdot \left(\frac{s-1}{\sum s}\right)ds\;\cdot w_{i}+\frac{s}{\sum s}\cdot w^{\prime },\;{\frac{1}{w}}_{i}\neq 0_{i}. \end{array}\right. \end{array}$$

Among them, the weight 1/*w*_*i*_ is included. Then, five samples are selected from each class, and the students who meet the requirements are queued, sorted according to their date of birth, and selected by a random equidistant sampling method. A total of 60 students were selected from each grade for investigation, 250 students were selected from each school, and 1752 students were selected as special investigation objects.

The teaching content and credit investigation: College students' physical education teaching system investigates the teaching content and credits, and operates according to the system instructions. Before operating the system, give 2.5 h explanation and 0.5 h operation practice to relevant personnel. Each operation is carried out by more than 2 teachers, one of whom has more than 2 years of teaching experience. Investigate students' teaching content and credits. The teaching contents and credits were investigated for 3 times, and the minimum and maximum values were eliminated, and the average values were taken. Among them, the credit survey is divided into units with an accuracy of 0.1 points. The survey grade of teaching content is unit, and the accuracy is 0.1. Adopt the standards of the Academic Affairs Office: grade, gender, teaching effect score, less than 25 points are poor; credit less than 45 is the difference; 25∼50 is medium; Credits of 45∼75 are medium. Assuming that the teaching score is *z*_*i*_, the analysis index is *x*_*i*_, the reference median is *m*_*i*_ , and the survey requirement is*c*_*i*_; the final score *Z* is calculated as shown in the following:

(2) $$\begin{array}{c} \left\{\begin{array}{c} Z=\sum \frac{\left(x_{i}-z_{i}\right)-m_{i}^{\prime \prime }}{c_{i}},\;c_{i}=0,\\ Z^{\prime }=\left(x_{i}-z_{i}\right)\cdot \sum \frac{\left(x_{i}-z_{i}\right)\prime -m_{i}^{\prime \prime }}{c_{i}^{\prime }},\;c_{i}\neq 0. \end{array}\right. \end{array}$$

The measurement of teaching effect: Everymonth, students are organized to evaluate the teaching effect of teachers, and the students' union of colleges and universities organizes learning. The system used is the existing online teaching system of colleges and universities. According to the investigation requirements in the research of “Methods for College Students' Physical Education,” the teaching effect scores of less than 25 are poor, 25∼60 are medium, 60∼80 are good, and 80∼100 are excellent. Because the survey object is the same university, the influence of neglected majors on the survey results is used.

The questionnaire survey refers to the relevant research materials of the Academic Affairs Office and combines the teaching characteristics of various majors; the questionnaire of students' satisfaction is designed. The contents include students' basic situation survey, satisfaction survey, and parents' satisfaction survey. It involves students' own basic situation, teaching responsibility, scientific teaching, and special credits; physical education knowledge of students' parents; reconstruction survey was added to the evaluation questionnaire, and the students' on-time class situation was counted..

## 3. Results

### 3.1. Statistical Analysis

Adopt the physical education system of the Ministry of Education to input, clean up, and calculate the data. The results of continuous variables $\bar{x}\pm s$ were expressed, the mean value between grades was compared by variance analysis, and the rate was compared by chi-square test.

### 3.2. General Teaching Materials

1003 male students (51.1%) and 961 female students (48.9%) were investigated. The ratio of male to female is 104 : 100. The gender and grade distribution of college students are shown in Table 2, and there is no significant difference in gender among grade groups (*P* < 0.05).

Among them, the third item in Table 2 is the number of satisfied people and the satisfaction rate. The satisfaction rate of graduate students is higher, followed by the satisfaction rate of freshmen. The satisfaction rate of men is higher than that of women. There is no difference in the satisfaction rate between college students and graduate students, but there are differences in the satisfaction rate between college students and graduate students. There is no significant difference in physical education teaching content and teaching methods. Therefore, there is no significant difference in gender, educational background, teaching content, and teaching methods among the research objects of this paper, which can be compared by statistics. In addition, the information obtained by the subjects in Table 2 is publicly obtained, which is also agreed upon by the investigators.

### 3.3. Status of Physical Education Teaching Content

There are 1452 valid data in the teaching content, and the average teaching content is 9.8 ± 1.4 points, and the average credit is 48.0 ± 2.9 points, as shown in Table 3.

The rates of poor teaching content, reexamination, and make-up examination of college students were 2.8%, 9.0%, and 10.1%, respectively, which had no significant difference from the survey of students of the same age (*P* > 0.05), but had a significant difference with the survey of other areas (*P* < 0.05). There was a statistical difference in the complaint rate among the three grades. With the increase in grades, the complaint rate increased (*P* < 0.05). There was no significant difference with the survey of students of the same age (*P* > 0.05), but there was a significant difference with the survey of students of the same age in other regions (*P* < 0.05). The *Z* score and complaint rate of college students in each grade group are shown in Tables 3 and 4.

It can be seen from Table 4 that the observation group is significantly better than the control group in terms of grade and teaching effect, the satisfaction grade of graduate students is significantly better than that of college students, and the average satisfaction grade and teaching effect of the observation group are better than that of the control group, and there are significant differences. There is no significant difference in gender between the observation group and the control group, and there is no significant difference in gender between college students and graduate students. There is no significant difference in gender between the average results of the observation group and the average results of the control group, so there is no significant difference in gender between the two groups of researchers. Although the overall results of the observation group and the control group have no significant difference, there are significant differences in the average results, which shows that satisfaction grade and teaching effect are the main influencing factors of college students' satisfaction and also the main factors affecting *Z* score.

In order to improve the accuracy in Table 5, change all data in the table to 0.1. At the same time, the accuracy of the data in Table 4 is 0.1 bits, which meets the statistical requirements of the data in this questionnaire. The data in Table 4 show that the satisfaction of the observation group is significantly better than that of the control group. Graduate students' satisfaction is higher than that of college students, and there are also significant differences. In addition, the overall satisfaction of the whole school, the observation group is also better than the control group. Therefore, the overall satisfaction of the observation group is significantly better than that of the control group.

### 3.4. Physical Education Teaching Effect and Physical Education Teaching Cognition

The average awareness of physical education of college students is 52.0%, among which the awareness of physical education is 41.0%, the awareness of comparative physical education is 11.1%, and the awareness of extraordinary physical education is 0.9%, as shown in Table 6.

As can be seen from Table 6, low cognition, medium cognition, and high cognition are obvious in undergraduates, while high cognition has no statistical significance among grades. Physical education awareness is particularly important for postgraduates.

### 3.5. Factors Affecting Satisfaction

The factors with differences in the above table are analyzed by logistics, and the results in Table 7 are obtained.

It can be seen from Table 7 that grade, gender, cognition, credit, sense of responsibility, and teaching content are all factors affecting college students' satisfaction. Among them, restudy, cognition, grade, credit, and make-up test rates are the main influencing factors that directly affect the satisfaction of college physical education. The influence degree of different factors is shown in Figure 2.

As can be seen from Figure 2, there are many factors that affect more than 15%, accounting for about 20%, so the influencing factors analyzed in this paper are basically consistent with the actual monitoring results. As can be seen from Figure 2, there are many factors affecting the grade from 1 to 15, accounting for about 65%, and the influencing factors >15% account for about 45%. This shows that the influencing factors of satisfaction have a small influence level, and there are few factors that have more influence. At the same time, it also shows that different influencing factors have the same importance for satisfaction, so physical education should pay attention to each influencing factor and make comprehensive improvements on physical education. The contents in Table 7 show that the OR values of different influencing factors are the same, and cognition and satisfaction levels are the main influencing factors, which are also the factors with greater influence. Therefore, the results in Figure 2 verify the results in Table 7.

## 4. Discussion

The results of this study show that the complaint rate of college students in the study group and the awareness of physical education teaching is higher, while the teaching effect of undergraduate and graduate students is better. However, the teaching contents and credits of different grades in the study group are consistent with those in the control group.

### 4.1. Research on the Factors of Satisfaction Rate and Cognition

The undergraduate course is the key period for students to carry out physical education. The results of this paper show that the reeducation in undergraduate and graduate students shows a trend of rising first and then falling, and the awareness of physical education in low, middle and high undergraduate and graduate students is higher than that of the control group, with significant differences, but lower than that of the research group. Postgraduates are the key period of cognitive improvement, and the reeducation in this grade is relatively high, which shows that college students have serious problems in physical education reeducation. At the same time, in the study group of undergraduates, the graduate stage of the rerepair rate is lower than the control group, and there is still a difference with the control group, which further shows that the rerepair rate of the control group is higher, indicating that the rerepair rate is the main factor affecting satisfaction. The survey shows that the college students' awareness of physical education is over 40%, which is still a serious cognitive problem, Pulido-Gil et al. [6]. The research shows that the awareness of physical education among undergraduate students is 42.2%, which is higher than that of graduate students (32.4%), Patria [7]. The way of “satisfaction of physical education + physical education” can be adopted. With the increase of physical education teaching time, the rerepair rate of graduate students and undergraduate students will decline, which indicates that extending teaching time is conducive to reducing the rerepair rate of college students, which is consistent with the existing report conclusion, Mergulhao et al. [8]. The investigation in Northeast China Luo et al. [9], Southeast China Liu et al. [10], West China, and other places also shows that high awareness of physical education can significantly reduce students' restudy rate Liu and Zhuang [11], so it is very important to carry out effective physical education, Ji et al. [12], which can improve the physical education effect of college students, Hamilton et al. [13]. It is the key to further developing targeted physical education for college students.

### 4.2. Study on the Factors of Failure Rate and Awareness Rate

The survey results of college students show that the failure rate is 9%, which is lower than the baseline survey of 9.4%, but it does not reach the goal that the make-up examination rate of college students is less than 5% in the Physical Education Standards for College Students. The results of this study show that there is a significant difference between the make-up examination rate of undergraduate and graduate students and the control group. The above-mentioned problems may be related to the rationality and unreasonable content structure of physical education teaching for college students, which are less than 20%. Most parents of college students do not know about college physical education, and the awareness rate is only 12.4%, Gosalbez-Carpena et al. [14]. Therefore, it is the top priority of Qinghai people's work to increase the publicity of physical education knowledge for parents of college students. At the same time, the survey data of college students show that insufficient cognition will affect college physical education, and the make-up examination rate is 13.4%, which is higher than the current national average.

### 4.3. The Influence of Make-Up Test Rate

The results of this study show that the make-up examination rate of undergraduate and graduate students has dropped significantly, which is consistent with that of the control group. The reasons for the above problems are related to the gender, family, and age of college students. Because freshmen do not understand physical education, they will be tired of learning. Because of their own cognitive limitations, they often give up physical education. According to statistics, 50.3% of parents still insist on letting students take physical education, while the rest of the parents can still insist on letting their children make up the exam although they have no clear cognition Gashaye et al. [15]. According to the survey data, the attendance rate of college students in physical education is 95.2%, and the overall rate of attending classes on time is 44.2%, indicating that the make-up examination rate is also an important indicator affecting satisfaction.

### 4.4. The Significance of Investigating the Influencing Factors of Satisfaction

The results of this paper show that students with high satisfaction in physical education teaching have a lower complaint rate, awareness of physical education teaching and card supplement rate, and the teaching content and credits have been improved, which shows that satisfaction in physical education teaching is of great significance to the improvement of physical education teaching level. However, in this report, there are differences between undergraduate and graduate students' make-up examination rate and physical education awareness and the control group. The above reasons, on the one hand, are due to students' cognition of physical education, which cannot be changed for the time being. On the other hand, due to the reasonable teaching content, the satisfaction of physical education is not high, de Vinaspre-Hernandez et al. [16]. Some scholars believe that although college students have been studied and their parents have improved their knowledge of physical education, they still lack relevant cognition. Therefore, teachers should strengthen the propaganda of physical education knowledge, popularize the influence of physical education on students' physical fitness, Conde-Pipo et al. [17], help them change their cognition of physical education, and ensure the level of physical education and teachers' content Caponnetto et al. [18]. In a word, aiming at the influencing factors of physical education satisfaction Burns and Struessel [19], we should effectively reduce the incidence of make-up examination, reexamination, and unreasonable teaching content, vigorously publicize physical education knowledge, improve students' satisfaction with physical education, and realize the quality education of college physical education, Behzadnia et al. [20].

## 5. Conclusion

Satisfaction degree is an important index to evaluate physical education teaching content, and satisfaction degree is affected by many factors, so we should find out the influencing factors of satisfaction degree by statistical methods to provide support for the formulation of teaching strategies. Through statistical methods, this paper finds that content rationality, make-up test rate, Bean et al. [21], retest rate, complaint rate, and sense of responsibility are the main factors affecting satisfaction. Rationality and sense of responsibility are the factors with deep influence, while other factors are the factors with less influence. In addition, there are significant differences in the main influencing factors between college students and graduate students, Bartosiewicz et al. [22], but there is no difference between college students and graduate students. There was a significant difference between the average results of the control group and the observation group, but there was no significant difference in the results of the whole school. Therefore, the above-mentioned factors are the main factors affecting the satisfaction of physical education Badura-Brzoza et al. [23]. To improve the level of physical education, we should analyze the above-mentioned factors in a left-handed and comprehensive way. The results of this study are still insufficient. The correlation between the influencing factors, the independence of factors Al-Mulla and Mahfoud [24], and the impact of the increase of research factors on satisfaction are in-depth analyses. In future research, we will start from the above aspects to improve the depth of research.

## Figures and Tables

**Figure 1:** Influence degree of different influencing factors.

**Figure 2:** Influence degree of different factors.

**Table 1:** Influencing factors of college physical education.

	Grade		Gender	
	Undergraduate	Master's degree	Male	Female
Content	13.2	312	6.11	1.73
Satisfaction rate	13.2	721	8.32	1.96
Make-up rate	15.2	121	3.38	2.58
Complexity	23.2	22.1	4.13	1.13
Others	14.2	81.3	2.15	1.18

**Table 2:** General teaching materials.

Variable	Total number of cases	Total number of cases	Satisfaction rate (%)	*X * ^*2*^
Grade				
Specialist	641	542	443 (69.1)	0.672
Undergraduate	541	480	389 (71.9)	
Master's degree	749	661	535 (80.9)	

Gender				
Male	984	858	702 (71.3)	0.723
Female	947	825	665 (70.2)	

Grade				0.778
Freshman year	256	234	221 (94.4)	
Sophomore year	282	276	254 (92)	
Junior year	278	265	254 (95.8)	
Senior year	292	287	278 (92.9)	
Research 1	227	253	244 (92.4)	
Research 2	284	272	225 (92)	
Research 3	305	298	282 (94.2)	

Achievement				0.892
0∼45	253	242	239 (99.5)	
45∼80	272	222	258 (99.4)	
80∼100	235	232	229 (99.4)	

Sports content				0.782
Special	489	472	422 (94.8)	
Two items	498	482	442 (94.9)	
Triple	482	442	428 (99.2)	
More than three items	495	483	442 (94.4)	

Learning style				
Normal	984	948	924 (98.9)	
Reconstruct	944	924	953 (98.2)	

**Table 3:** Test results of credits and teaching contents of each grade group.

Grade	Teaching content (grade)	Credits (points)
	($\bar{x}\pm s$)	($\bar{x}\pm s$)
Undergraduate	8.5 ± 1.3^ab^	41.4 ± 4.9 ^ab^
Control group	8.4 ± 0.1^b^	40.2 ± 3.1^b^
Research group	4.2 ± 0.2	40.2 ± 2.4
Graduate student	9.4 ± 1.3 ^ab^	44.8 ± 4.4 ^ab^
Control group	9.2 ± 0.9^b^	44.4 ± 3.8^b^
Research group	8.3 ± 0.2	40.8 ± 3.1
The whole school	10.9 ± 1.5 ^ab^	83.2 ± 4.2 ^ab^
Control group	10.3 ± 0.9^b^	82.1 ± 3.1^b^
Research group	8.9 ± 0.8	80.2 ± 3.8
Average	9.8 ± 1.4 ^ab^	48.0 ± 2.9 ^ab^
Control group	9.4 ± 1.2^b^	44.1 ± 5.2^b^
Research group	8.8 ± 0.9	40.1 ± 5.3

Compared with the control group, ^*a*^*P* > 0.05; compared with the study group, ^*b*^*P* < 0.05.

**Table 4:** Average *Z* score of each grade group [*n*, ($\bar{x}\pm s$)].

Grade	Grade	Gender	Teaching effect
Undergraduate	0.14 ± 1.2^ab^	0.34 ± 1.4^ab^	0.28 ± 1.4^ab^
Control group	0.13 ± 0.9^b^	0.32 ± 0.9^b^	0.24 ± 0.3^b^
Research group	0.02 ± 0.24	0.29 ± 1.4	0.12 ± 0.4
Graduate student	0.22 ± −1.2^ab^	0.22 ± 1.4^ab^	0.33 ± 1.5^ab^
Control group	0.12 ± 0.9^b^	0.32 ± 1.4^b^	0.32 ± 1.2^b^
Research group	0.22 ± 0.22	0.12 ± 0.4	0.19 ± 0.5
The whole school	0.32 ± −1.1^ab^	0.83 ± 1.1^ab^	0.29 ± 1.4^ab^
Control group	0.31 ± 0.92^b^	0.23 ± 0.8^b^	0.22 ± 0.8^b^
Research group	0.23 ± 0.31	0.11 ± 0.9	0.12 ± 0.1
Average	0.23 ± 1.29^ab^	0.12 ± 1.2^ab^	0.32 ± 1.4^ab^
Control group	0.28 ± 0.92^b^	0.18 ± 0.5^b^	0.39 ± 1.3^b^
Research group	0.1 ± 1.14	0.03 ± 0.1	0.01 ± 0.4

Compared with the control group, ^*a*^*P* > 0.05; compared with the study group, ^*b*^*P* < 0.05.

**Table 5:** Comparison of complaint rates among different grade groups.

Variable	Undergraduate	Graduate student	The whole school
Poor teaching content (%)	42.1 ± 4.3^bc^	39.2 ± 4.5^ab^	39.3 ± 5.3^ab^
Control group	4.2^b^	2.4 ± 0.3^b^	5.1 ± 2.1^b^
Research group	9.2	8.9	2.3
Satisfaction rater (%)	45.3 ± 4.8^bc^	52.6 ± 9.9^ab^	24.6 ± 9.2^ab^
Control group	4.2^b^	9.4 ± 0.23^b^	8.9^b^
Research group	8.2	1.4 ± 0.2	10.2
Make-up examination rate (%)	201.3 ± 0.2^ab^	58.5 ± 11.1^ab^	25.2 ± 8.9 ^ab^
Control group	1.3 ± 0.1^b^	10.9 ± 0.52^b^	8.8^b^
Research group	1.8 ± 1.8	12.4	9.2 ± 0.32
Failure rate (%)	22 ± 3.8^ab^	14.7 ± 3.3 ^ab^	12.1 ± 2.2 ^ab^
Control group	3.2^b^	3.4^b^	2.3^b^
Research group	4.2 ± 1203	4.1	3.1
Elimination rate (%	4.2 ± 1.2 ^ab^	8.8 ± 1.5 ^ab^	9.2 ± 1.2 ^ab^
Control group	1.1^b^	1.2^b^	1.3^b^
Research group	2.1	2.2	2.8

Compared with the control group, ^*a*^*P* > 0.05; compared with the study group, ^*b*^*P* < 0.05.

**Table 6:** Physical education teaching effect and teaching awareness of each grade group.

Variable	Undergraduate	Graduate student	The whole school
Low awareness	254 ± 40.9^ab^	233 ± 43.9 ^ab^	284 ± 38.4 ^ab^
Control group	39.5^b^	42.3^b^	38.9^b^
Research group	4 ± 5.2	4 ± 9.2	4 ± 2.3
Moderate awareness	81 ± 12.9^ab^	39 ± 13.0 ^ab^	20 ± 8.1 ^ab^
Control group	12 ± 2.8^b^	12 ± 2.2^b^	8.0^b^
Research group	13 ± 4.2	11 ± 5.2	9.3
High awareness	53 ± 0.8 ^ab^	21 ± 1.1 ^ab^	2 ± 0.8 ^ab^
Control group	0.4^b^	1.0^b^	0.9^b^
Research group	1.2	1.3	1.1

Compared with the control group, ^*a*^*P* > 0.05; Compared with the study group, ^*b*^*P* < 0.05.

**Table 7:** Satisfaction analysis of influencing factors.

Influencing factors	B	OR	CI95%		*P*
			Upper limit	Lower limit	
Grade	112.24	41.14	2.12	12.24	0.01
Gender	19.18	8.12	8.12	91.18	0.02
Cognition	110.20	122.24	9.18	111.14	0.03
Credit	121.22	21.12	10.20	14.14	0.00
Responsibility	14.14	10.20	2.12	10.20	0.03
Teaching content	15.10	9.18	9.18	10.20	0.04
Failure rate	12.12	5.10	12.24	14.14	0.02
Satisfaction rate	112.24	8.12	12.24	15.10	0.04
Complaint rate	34.14	4.14	10.20	12.24	0.04
Make-up rate	19.18	11.22	10.20	11.18	0.00

## Data Availability

The data used to support the findings of this study are available from the corresponding author upon request.
